The article "Analysis and Simulation of Fractional Order Smoking Epidemic Model" was published in 2022. Journal: Comput Math Methods Med.

# Analysis and Simulation of Fractional Order Smoking Epidemic Model

**DOI:** 10.1155/2022/9683187

**Published:** 2022-05-20

**Authors:** Aqeel Ahmad, Muhammad Farman, Abdul Ghafar, Mustafa Inc, Mohammad Ozair Ahmad, Ndolane Sene

**Affiliations:** ^1^Department of Mathematics, Ghazi University, DG Khan, Pakistan; ^2^Department of Mathematics and Statistics, University of Lahore, Lahore 54590, Pakistan; ^3^Department of Computer Engineering, Biruni University, Istanbul, Turkey; ^4^Department of Mathematics, Science Faculty, Firat University, Elazig, Turkey; ^5^Department of Medical Research, China Medical University, Taichung, Taiwan; ^6^Laboratoire Lmdan, Departement De Mathematiques De Decision, Facultíe des Sciences Economiques et Gestion, Universite Cheikh Anta Diop De Dakar, BP 5683 Dakar Fann, Senegal

## Abstract

In recent years, there are many new definitions that were proposed related to fractional derivatives, and with the help of these definitions, mathematical models were established to overcome the various real-life problems. The true purpose of the current work is to develop and analyze Atangana-Baleanu (AB) with Mittag-Leffler kernel and Atangana-Toufik method (ATM) of fractional derivative model for the Smoking epidemic. Qualitative analysis has been made to `verify the steady state. Stability analysis has been made using self-mapping and Banach space as well as fractional system is analyzed locally and globally by using first derivative of Lyapunov. Also derive a unique solution for fractional-order model which is a new approach for such type of biological models. A few numerical simulations are done by using the given method of fractional order to explain and support the theoretical results.

## 1. Introduction

Mathematics was firstly used in biology in the twelfth century when Fibonacci used his popular Fibonacci series to explain a growing population. Daniel Bernoulli used mathematics to describe the effect of small pox. The term biological mathematics was primarily used by Johannes Reinke in 1901. It is aimed at the mathematical image and modeling of biological processes. It is also used to recognize phenomena in the living organism. Bio math has made major progress during the last few decades, and this progress will continue in upcoming decades. Math has played a large role in natural science but now it also will be more useful in biology. We should teach basic concepts of bio math at early stages. The basic steps in mathematical biology are few. The initial step is to explain the biological process and raise a question about the basics. The second step is to build up a mathematical model that represents the underlying biological process. The 3rd step is to apply the method and concepts of math to obtain predictions about the model. The last step is to check whether this prediction answers the raised questions. After this, anyone can further explore the biological question by using mathematical models [1].

The article "Analysis and Simulation of Fractional Order Smoking Epidemic Model" was published in 2022. Journal: Comput Math Methods Med.

Now in the modern world, tobacco smoke is the most inhaled substance. Tobacco is made by mixing its agricultural form with many substances. The smoke is inhaled through the lungs. The most dangerous epidemic in the world is the smoking epidemic. Due to smoking 50% of its users died. Every year, about 60 million people die due to smoking. During the last few decades, there has been a huge boost in deaths. The death rate will rise thrice annually in 2030, almost seventy percent is in developing countries. According to WHO, 10 million people will die due to smoking. As compared to other diseases, the death ratio is higher than all. The person who uses tobacco dies 14 years earlier than someone who does not smoke [2]. Tobacco smoking is the major reason for cancer and another disease. About 70% of people died due to tobacco-related diseases in developing countries [3]. Three million people died due to smoking yearly.

Nowadays, smoking is the most dangerous habit. The heart attack ratio is 70 percent more than a nonsmoker. There are 900 million men smokers and 200 women smokers in the world. After every 6 seconds, there is a death due to smoking. Smoking is a major cause of lung and heart attack in the world. Due to smoking, the chances of other diseases like heart attack, stroke, especially lung cancer, throat, mouth, esophagus, and pancreas are increased. Tobacco causes many tissue-related diseases. Tobacco smoke is a mixture of several toxic gases. It includes 98 of which are linked with an increased risk of cardiovascular disease, 69 of which are known to be carcinogenic. Daily, a smoker takes 1 or 2 milligrams of nicotine per cigarette. Thus, if a person smokes 5 cigarettes, it takes at least 5-10 milligrams of nicotine. The effect of smoking is not limited to the person who but also adverse effects for other people. It causes 22% of death annually.

The chemical composition of tobacco varies according to the environment. These leaves are mixed with many chemicals. Tobacco smoke contains a large number of different chemicals such as benzopyrene, NNK, aldehydes, carbon monoxide, hydrogen cyanide, phenol, nicotine, and harmala alkoids. The radioactive element polonium 210 is also occurring in tobacco. There are almost 4 thousand noxious substances in smoke which is the main reason for cancer [4, 5]. The chemical composition of smoke depends on puff frequency and other materials. Nicotine is the main issue for disturbing the nervous system, rise in heartbeat, raising blood pressure, and shrinking the small blood vessels which are the main basis of wrinkles. The amount of oxygen decreased in the lungs due to carbon monoxide (CO). The natural lungs cleaner that is minuscule hairs is destroyed by hydrogen cyanide. Lead, nickel arsenic, and cadmium are also present in smoke. Some pesticides like DDT are also found in smoke. The major reason for skin and lung cancer is a toxic chemical that is present in smoke. 10 million deaths will occur in the 20^th^ century and 1 billion in the 21st century due to smoking [6]. Cigarette smoking affects human fertility badly [7].

The article "Analysis and Simulation of Fractional Order Smoking Epidemic Model" was published in 2022. Journal: Comput Math Methods Med.

The generalization of classical calculus is called fractional calculus which is concerned with the operation of integration and differentiation of fractional order. In the 19th century, fractional calculus mathematicians introduced fractional differential equations, fractional dynamics, and fractional geometry. Fractional calculus is used in almost every field of science. It is used to model physical as well as engineering processes. In many cases, standard mathematical models of integer order do not work properly. Due to this reason, fractional calculus made a major contribution to the field of mechanics, chemistry, biology, and image processing. By using fractional calculus, several physical problems are solved. By using integer-order derivatives, the system shows many problems such as history and nonlocal effects. Primarily, all the studies were dependent on Caputo fractional-order and Reimann Liouville fractional (RLF) derivatives. Nowadays, it has been highlighted that these derivatives have the issue, and the issue is they have a singular kernel. That is the reason so many new definitions were presented in the studies [8–16]. These new definitions were very impactful because they have nonsingular kernels which are according to their needs. Caputo fractional derivatives [17], the Caputo-Fabrizio derivative [11], and AB [18] fractional derivative have differed from each other only because Caputo is defined by a power law, Fabrizio defined by using exponential decay law, and AB defined by ML law. Tateishi et al. describe the role of fractional time operator derivative in a study of anomalous diffusion [12]. With the help of analytical techniques, Bulut et al. deliberate the role of differential equations of arbitrary order [19]. The key concepts of fractional differential equations and their application are explained by Kilbas et al. [20]. Atangana and Koca examined the Keller-Segel model about a fractional derivative having a nonsingular kernel [21]. Fractional logistic maps are newly introduced by Huang et al. [22]. Zaman studied the qualitative response of the dynamics of giving up smoking [23]. The giving up smoking model linked with Caputo fractional derivative is a probe by Singh et al. [24].

The article "Analysis and Simulation of Fractional Order Smoking Epidemic Model" was published in 2022. Journal: Comput Math Methods Med.

Numerous studies identified sociodemographic, environmental, and behavioral risk factors such as age, sex, occupations, indoor air pollutions, smoking, and alcohol consumption [25–27] as being associated with the development of TB in humans. In [28], a simple model for the effect of tobacco smoking in the in-host dynamics of HIV is formulated with the aim of studying how tobacco smoking affects HIV in-host dynamics. Zoonotic tuberculosis (zTB) knowledge, prevention, and control practices via a survey in Bangladesh considering impact of smoking are also in [29].

In this work, we get the approximate solutions of the fractional smoking model by using the Atangana-Toufik method.

## 2. Basic Concepts of Fractional Operators

**Definition 1 .**

For a function *g*(*t*) ∈ *W*_2_^1^(0, 1), *b* > *a* and *σ* ∈ [0, 1], the definition of AB derivative in the Caputo sense is given by

(1) Dtσ0ABCgt=ABσ1−σ∫0tddτgτMσ−σ1−σt−τσdτ, n−1<σ<n,

where

(2) $$\begin{array}{c} \text{AB}\left(\sigma \right)=1-\sigma +\frac{\sigma }{\Gamma \left(\sigma \right)}. \end{array}$$

By using ST for (1), we obtain

(3) STDtσ0ABCgts=qσ1−σσΓσ+1Mσ−11−σVσ×STgt−g0.

**Definition 2 .**

The Laplace transform (LT) of the Caputo fractional derivative of a function  *g*(*t*) of order *σ* > 0 is defined as

(4) LDtσ0Cgt=sσgs−∑σ=0n−1gσ0sσ−v−1.

**Definition 3 .**

The LT of the function *t*^*σ*_1_−1^*E*_*σ*,*σ*_1__(±*μt*^*σ*^) is defined as

(5) $$\begin{array}{c} L\left[t^{\sigma_{1}-1}E_{\sigma ,\sigma_{1}}\left(\pm \mu t^{\sigma }\right)\right]=\frac{s^{\sigma -\sigma_{1}}}{s^{\sigma }\mp \mu }, \end{array}$$

where *E*_*σ*,*σ*_1__  is the two-parameter ML function with  *σ*, *σ*_1_ > 0. Further, the ML function satisfies the following equation [17].

(6) $$\begin{array}{c} E_{\sigma ,\sigma_{1}}\left(f\right)=fE_{\sigma ,\sigma +\sigma_{1}}\left(f\right)+\frac{1}{\Gamma \left(\sigma_{1}\right)}. \end{array}$$

**Definition 4 .**

Suppose that *g*(*t*)  is continuous on an open interval (*a*, *b*), then the fractal-fractional integral of *g*(*t*)  of order *σ* having ML type kernel and given by

(7) JFFM0,tσ,σ1gt=σσ1ABσΓσ1∫0tsσ1−1gst−sσds+σ11−σtσ1−1gtABσ.

## 3. Model Formulation

We will study the giving up smoking model for overall population at time *t*. We separate the population into 5 groups, potential smokers *P*(*t*), occasional smokers *L*(*t*), heavy smokers *S*(*t*), temporary quitters *Q*(*t*), and smokers who quit permanently *R*(*t*) specified by *T*(*t*) = *P*(*t*) + *L*(*t*) + *S*(*t*) + *Q*(*t*) + *R*(*t*). Due to smoking, the chances of other diseases like heart attack, stroke, especially lung cancer, throat, mouth, esophagus, and pancreas are increased [24]. The model is developed as follows

(8) $$\begin{array}{c} \frac{dP}{dt}=a\left(1-P\right)-bPS, \end{array}$$

(9) $$\begin{array}{c} \frac{dL}{dt}=-aL+bPL-cLS, \end{array}$$

(10) $$\begin{array}{c} \frac{dS}{dt}=-\left(a+d\right)+cLS+fQ, \end{array}$$

(11) $$\begin{array}{c} \frac{dQ}{dt}=-\left(a+f\right)Q+d\left(1-e\right)S, \end{array}$$

(12) $$\begin{array}{c} \frac{dR}{dt}=-aR+edS. \end{array}$$

With the initial conditions

(13) $$\begin{array}{c} P\left(0\right)=\delta_{1}, \end{array}$$

(14) $$\begin{array}{c} L\left(0\right)=\delta_{2}, \end{array}$$

(15) $$\begin{array}{c} S\left(0\right)=\delta_{3}, \end{array}$$

(16) $$\begin{array}{c} Q\left(0\right)=\delta_{4}, \end{array}$$

(17) $$\begin{array}{c} R\left(0\right)=\delta_{5}. \end{array}$$

The rate of change between potential smoker and occasional smokers is represented by *b*, *a* represents the rate of natural death, the rate of occasional smoker and temporary smokers by *c*, the rate of change between quitters and smoker is shown by *f*, the rate of giving up smoking is shown by *d*, fraction of temporary giving up smoker is represented by (1 − *e*) (at the rate of *d*), *e* shows the remaining fraction of smokers who give up smoking forever (at a rate *d*).

The article "Analysis and Simulation of Fractional Order Smoking Epidemic Model" was published in 2022. Journal: Comput Math Methods Med.

## 4. Qualitative Analysis

By substituting the values of parameters in given system of differential equations and the rate of change with respect to time is zero, we get

(18) $$\begin{array}{c} a\left(1-P\right)-bPS=0, \end{array}$$

(19) $$\begin{array}{c} -aL+bPS-cLS=0, \end{array}$$

(20) $$\begin{array}{c} -\left(a+d\right)S+cLS+fQ=0, \end{array}$$

(21) $$\begin{array}{c} -\left(a+f\right)Q+d\left(1-e\right)S=0, \end{array}$$

(22) $$\begin{array}{c} -aR+edS=0. \end{array}$$

By simplifying the above equations, we get disease-free equilibrium, denoted by *E*_0_, i.e., *E*_0_ = (1, 0, 0, 0, 0).

Endemic equilibrium is found in terms of one of the infected compartment, denoted by *E*_1_, i.e., *E*_1_ = (*P*^∗^, *L*^∗^, *S*^∗^, *Q*^∗^, *R*^∗^) where *P*^∗^ = *a*/*a* + *bS*^∗^, *L*^∗^ = *ab*/(*a* + *bS*^∗^)(*a* + *cS*^∗^), *Q*^∗^ = *d*(1 − *e*)*S*^∗^/*a* + *f*, *R*^∗^ = *edS*^∗^/*a*.

### 4.1. Stability Analysis and Reproductive Number

It is important to find the verge conditions to check the status of population, whether the disease persist or dies out. In case of disease free equilibrium point, *R*_0_ < 1, which shows that the disease will die out. In case of endemic equilibrium, *R*_0_ > 1. Consider the Jacobian matrix (JM) as

(23) $$\begin{array}{c} J=\left[\begin{array}{ccccc} -a-bS & 0 & -bP & 0 & 0\\ bS & -a-cS & bP-cL & 0 & 0\\ 0 & cS & -a-d+cL & f & 0\\ 0 & 0 & d\left(1-e\right) & -a-f & 0\\ 0 & 0 & ed & 0 & -a \end{array}\right]. \end{array}$$

Since the JM is *J* = *F* − *V* where

We know that *K* = FV^−1^ and using the relation |*K* − *λI*| = 0 solving on mathematica for the Eigenvalue *λ*, which represents the reproductive number *R*_0_, i.e.,

(24) $$\begin{array}{c} R_{0}=\frac{df\left(1-e\right)}{\left(a+d\right)\left(a+f\right)}. \end{array}$$

Hence, *R*_0_ = 0.431034 < 1, according to the given parameter values.

The article "Analysis and Simulation of Fractional Order Smoking Epidemic Model" was published in 2022. Journal: Comput Math Methods Med.

**Theorem 1 .**

The disease free equilibrium *E*_0_  is locally asymptotically stable for *R*_0_ < 1, if Re(*λ*) < 0, otherwise, unstable.

**Proof**

*E*_0_ of the given system is locally asymptotically stable if Re(*λ*) < 0 where *λ* can be evaluated from the relation |*J*_0_ − *λ*I| = 0.

By using the relation |*J*_0_ − *λ*I| = 0, we get. Re(*λ*) as

(25) $$\begin{array}{c} \lambda_{1}=-a,\lambda_{2}=\frac{1}{2}\left[-2a-d-f-\sqrt{d^{2}+2df-4def+f^{2}}\right]<0, \end{array}$$

(26) $$\begin{array}{c} \lambda_{3}=\frac{1}{2}\left[-2\text{a}-\text{d}-\text{f}+\sqrt{{\text{d}}^{2}+2\text{df}-4\text{def}+{\text{f}}^{2}}\right]<0\lambda_{1}. \end{array}$$

All the Eigenvalues are negative real parts which represent that the given system is locally asymptotically stable.

**Theorem 2 .**

When the reproductive number *R*_0_ > 1, the endemic equilibrium points *E*_1_ of the PLSQR model is globally asymptotically stable.

**Proof**

The Lyapunov function can be written as

(27) $$\begin{array}{c} M\left(P^{*},L^{*},S^{*},Q^{*},R^{*}\right)=\left(P-P^{*}-P^{*}\log\frac{P^{*}}{P}\right)+\left(L-L^{*}-L^{*}\log\frac{L^{*}}{L}\right)+\left(S-S^{*}-S^{*}\log\frac{S^{*}}{S}\right)+\left(Q-Q^{*}-Q^{*}\log\frac{Q^{*}}{Q}\right)+\left(R-R^{*}-R^{*}\log\frac{R^{*}}{R}\right). \end{array}$$

Therefore, applying the derivative respect to *t* on both sides yields

(28) $$\begin{array}{c} \frac{dM}{dt}=\dot{M}=\left(\frac{P-P^{*}}{P}\right)\dot{P}+\left(\frac{L-L^{*}}{L}\right)\dot{L}+\left(\frac{S-S^{*}}{S}\right)\dot{S}+\left(\frac{Q-Q^{*}}{Q}\right)\dot{Q}+\left(\frac{R-R^{*}}{R}\right)\dot{R}. \end{array}$$

Now, we can write their values for derivatives as follows

(29) $$\begin{array}{c} \frac{dM}{dt}=\dot{M}=\left(\frac{P-P^{*}}{P}\right)\left(a\left(1-P\right)-bPS\right)+\left(\frac{L-L^{*}}{L}\right)\left(-aL+bPS-cLS\right)+\left(\frac{S-S^{*}}{S}\right)\left(-\left(a+d\right)S+cLS+fQ\right)+\left(\frac{Q-Q^{*}}{Q}\right)\left(-\left(a+f\right)Q+d\left(1-e\right)S\right)+\left(\frac{R-R^{*}}{R}\right)\left(-aR+edS\right). \end{array}$$

Putting *P* = *P* − *P*^∗^,  *L* = *L* − *L*^∗^,  *S* = *S* − *S*^∗^,  *Q* = *Q* − *Q*^∗^,  *R* = *R* − *R*^∗^ leads to

(30) $$\begin{array}{c} \frac{dM}{dt}=\left(\frac{P-P^{*}}{P}\right)\left(a\left(1-\left(P-P^{*}\right)\right)-b\left(P-P^{*}\right)\left(S-S^{*}\right)\right)+\left(\frac{L-L^{*}}{L}\right)\left(-a\left(L-L^{*}\right)+b\left(P-P^{*}\right)\left(S-S^{*}\right)-c\left(L-L^{*}\right)\left(S-S^{*}\right)\right)+\left(\frac{S-S^{*}}{S}\right)\left(-\left(a+d\right)\left(S-S^{*}\right)+c\left(L-L^{*}\right)\left(S-S^{*}\right)+f\left(Q-Q^{*}\right)\right)+\left(\frac{Q-Q^{*}}{Q}\right)\left(-\left(a+f\right)\left(Q-Q^{*}\right)+d\left(1-e\right)\left(S-S^{*}\right)\right)+\left(\frac{R-R^{*}}{R}\right)\left(-a\left(R-R^{*}\right)+ed\left(S-S^{*}\right)\right). \end{array}$$

We can organize the above as follows

(31) $$\begin{array}{c} \frac{dM}{dt}=a-\left(\frac{P^{*}}{P}\right)a-\frac{1}{P}{\left(P-P^{*}\right)}^{2}-\frac{b}{P}{\left(P-P^{*}\right)}^{2}\left(S\right)+\frac{b}{P}{\left(P-P^{*}\right)}^{2}\left(S^{*}\right)-\frac{a}{L}{\left(L-L^{*}\right)}^{2}+bPS-{bP}^{*}S+bP^{*}S^{*}-bPS^{*}-\left(\frac{L^{*}}{L}\right)bPS+\left(\frac{L^{*}}{L}\right){bP}^{*}S-\;\left(\frac{L^{*}}{L}\right)bP^{*}S^{*}+\left(\frac{L^{*}}{L}\right)bPS^{*}-\frac{C}{L}{\left(L-L^{*}\right)}^{2}\left(S\right)+\frac{C}{L}{\left(L-L^{*}\right)}^{2}\left(S^{*}\right)-\frac{\left(a+d\right)}{S}{\left(S-S^{*}\right)}^{2}+\frac{c}{S}\left(L\right){\left(S-S^{*}\right)}^{2}-\frac{c}{S}\left(L^{*}\right){\left(S-S^{*}\right)}^{2}+f\left(Q\right)-f\left(Q^{*}\right)-\left(\frac{S^{*}}{S}\right)fQ+\left(\frac{S^{*}}{S}\right)fQ^{*}-\frac{\left(a+f\right)}{Q}{\left(Q-Q^{*}\right)}^{2}+d\left(1-e\right)\left(S\right)-d\left(1-e\right)\left(S^{*}\right)-d\left(1-e\right)\left(S\right)\left(\frac{Q^{*}}{Q}\right)+d\left(1-e\right)\left(S^{*}\right)\left(\frac{Q^{*}}{Q}\right)-\frac{a}{R}{\left(R-R^{*}\right)}^{2}+ed\left(S\right)-ed\left(S^{*}\right)-ed\left(S\right)\left(\frac{R^{*}}{R}\right)+ed\left(S^{*}\right)\left(\frac{R^{*}}{R}\right). \end{array}$$

To avoid the complexity, the above can be written as

(32) $$\begin{array}{c} \frac{dM}{dt}=\Sigma -\Omega , \end{array}$$

where

(33) $$\begin{array}{c} \Sigma =a+\frac{b}{P}{\left(P-P^{*}\right)}^{2}\left(S^{*}\right)+bPS+bP^{*}S^{*}+\left(\frac{L^{*}}{L}\right){bP}^{*}S+\left(\frac{L^{*}}{L}\right)bPS^{*}+\frac{C}{L}{\left(L-L^{*}\right)}^{2}\left(S^{*}\right)+\frac{c}{S}\left(L\right){\left(S-S^{*}\right)}^{2}+f+\left(\frac{S^{*}}{S}\right)fQ^{*}+d\left(1-e\right)\left(S\right)+d\left(1-e\right)\left(S^{*}\right)\left(\frac{Q^{*}}{Q}\right)+ed\left(S\right)+ed\left(S^{*}\right)\left(\frac{R^{*}}{R}\right), \end{array}$$

(34) $$\begin{array}{c} \Omega =\left(\frac{P^{*}}{P}\right)a+\frac{1}{P}{\left(P-P^{*}\right)}^{2}+\frac{b}{P}{\left(P-P^{*}\right)}^{2}\left(S\right)+\frac{a}{L}{\left(L-L^{*}\right)}^{2}+{bP}^{*}S+bPS^{*}+\left(\frac{L^{*}}{L}\right)bPS+\;\left(\frac{L^{*}}{L}\right)bP^{*}S^{*}+\frac{C}{L}{\left(L-L^{*}\right)}^{2}\left(S\right)+\frac{\left(a+d\right)}{S}{\left(S-S^{*}\right)}^{2}+\frac{c}{S}\left(L^{*}\right){\left(S-S^{*}\right)}^{2}+fQ^{*}+\left(\frac{S^{*}}{S}\right)fQ+\frac{\left(a+f\right)}{Q}{\left(Q-Q^{*}\right)}^{2}+d\left(1-e\right)\left(S^{*}\right)+d\left(1-e\right)\left(S\right)\left(\frac{Q^{*}}{Q}\right)+\frac{a}{R}{\left(R-R^{*}\right)}^{2}+ed\left(S^{*}\right)+ed\left(S\right)\left(\frac{R^{*}}{R}\right). \end{array}$$

It is concluded that if *Σ* < *Ω*, this yields, *dM*/*dt* < 0, however when, *P* = *P*^∗^, *L* = *L*^∗^, *S* = *S*^∗^, *Q* = *Q*^∗^, *R* = *R*^∗^

(35) $$\begin{array}{c} 0=\Sigma -\Omega \Rightarrow \frac{dM}{dt}=0. \end{array}$$

We can see that the largest compact invariant set for the suggested model in

(36) $$\begin{array}{c} \left\{\left(P^{*},L^{*},S^{*},Q^{*},R^{*}\right)\in \Gamma ;\frac{dM}{dt}=0\right\}, \end{array}$$

is the point {*E*_1_} the endemic equilibrium of the considered model. By the help of the Lasalles invariance concept, it follows that *E*_1_ is globally asymptotically stable in Γ if *Σ* < *Ω*.

The article "Analysis and Simulation of Fractional Order Smoking Epidemic Model" was published in 2022. Journal: Comput Math Methods Med.

## 5. Atangana-Baleanu Caputo Sense with Mittag-Leffler Kernel

By applying AB fractional derivative of order *σ* and *σ* ∈ (0, 1], into ML kernel, then, the system (8) becomes

(37) D0ABCtσP=a 1−P−bPS,

(38) DtσL=0ABC−aL+bPL−cLS,

(39) DtσS=0ABC−a+dS+cLS+fQ,

(40) DtσQ=0ABC−a+fQ+d1−eS,

(41) DtσR=0ABC−aR+edS.

The initial conditions associated with the system (37) are

(42) $$\begin{array}{c} P\left(0\right)=\delta_{1}, \end{array}$$

(43) $$\begin{array}{c} L\left(0\right)=\delta_{2}, \end{array}$$

(44) $$\begin{array}{c} S\left(0\right)=\delta_{3}, \end{array}$$

(45) $$\begin{array}{c} Q\left(0\right)=\delta_{4}, \end{array}$$

(46) $$\begin{array}{c} R\left(0\right)=\delta_{5}. \end{array}$$

We will discuss the numerical value of solution of system for different values of *ρ*. With the help of iterative method and the Padè approximation results are obtained.

We use the values of the parameters *a* = 0.04,  *b* = 0.23,  *c* = 0.3, *d* = 0.2,  *e* = 0.4, and *f* = 0.25. The initial conditions are given by *P* (0) = 0.60301,  *L* (0) = 0.24000,  *S* (0) = 0.10628, *Q*(0) = 0.03260, and *R*(0) = 0.01811.

Taking ST on both sides of (37), we get

(47) $$\begin{array}{c} \frac{q\left(\sigma \right)\sigma \Gamma \left(\sigma +1\right)}{1-\sigma }N_{\sigma }\left(-\frac{1}{1-\sigma }V^{\sigma }\right)\text{ST}\left\{P\left(t\right)-P\left(0\right)\right\}=\text{ST}\left[a\left(1-P\right)-bPS\right], \end{array}$$

(48) $$\begin{array}{c} \frac{q\left(\sigma \right)\sigma \Gamma \left(\sigma +1\right)}{1-\sigma }N_{\sigma }\left(-\frac{1}{1-\sigma }V^{\sigma }\right)\text{ST}\left\{L\left(t\right)-L\left(0\right)\right\}=\text{ST}\left[-aL+bPL-cLS\right], \end{array}$$

(49) $$\begin{array}{c} \frac{q\left(\sigma \right)\sigma \Gamma \left(\sigma +1\right)}{1-\sigma }N_{\sigma }\left(-\frac{1}{1-\sigma }V^{\sigma }\right)\text{ST}\left\{S\left(t\right)-S\left(0\right)\right\}=\text{ST}\left[-\left(a+d\right)S+cLS+fQ\right], \end{array}$$

(50) $$\begin{array}{c} \frac{q\left(\sigma \right)\sigma \Gamma \left(\sigma +1\right)}{1-\sigma }N_{\sigma }\left(-\frac{1}{1-\sigma }V^{\sigma }\right)\text{ST}\left\{Q\left(t\right)-Q\left(0\right)\right\}=\text{ST}\left[-\left(a+\text{f}\right)Q+d\left(1-e\right)S\right], \end{array}$$

(51) $$\begin{array}{c} \frac{q\left(\sigma \right)\sigma \Gamma \left(\sigma +1\right)}{1-\sigma }N_{\sigma }\left(-\frac{1}{1-\sigma }V^{\sigma }\right)\text{ST}\left\{R\left(t\right)-R\left(0\right)\right\}=\text{ST}\left[-aR+edS\right]. \end{array}$$

Rearranging, we get

(52) $$\begin{array}{c} \text{ST}\left(P\left(t\right)\right)=P\left(0\right)+\frac{1-\sigma }{q\left(\sigma \right)\sigma \Gamma \left(\sigma +1\right)N_{\sigma }\left(-\left(1/1-\sigma \right)V^{\sigma }\right)}\text{ST}\left[a\left(1-P\right)-bPS\right], \end{array}$$

(53) $$\begin{array}{c} \text{ST}\left(L\left(t\right)\right)=L\left(0\right)+\frac{1-\sigma }{q\left(\sigma \right)\sigma \Gamma \left(\sigma +1\right)N_{\sigma }\left(-\left(1/1-\sigma \right)V^{\sigma }\right)}\text{ST}\left[-aL+bPL-cLS\right], \end{array}$$

(54) $$\begin{array}{c} \text{ST}\left(S\left(t\right)\right)=S\left(0\right)+\frac{1-\sigma }{q\left(\sigma \right)\sigma \Gamma \left(\sigma +1\right)N_{\sigma }\left(-\left(1/1-\sigma \right)V^{\sigma }\right)}\text{ST}\left[-\left(a+d\right)S+cLS+fQ\right], \end{array}$$

(55) $$\begin{array}{c} \text{ST}\left(Q\left(t\right)\right)=Q\left(0\right)+\frac{1-\sigma }{q\left(\sigma \right)\sigma \Gamma \left(\sigma +1\right)N_{\sigma }\left(-\left(1/1-\sigma \right)V^{\sigma }\right)}\text{ST}\left[-\left(a+f\right)Q+d\left(1-e\right)S\right], \end{array}$$

(56) $$\begin{array}{c} \text{ST}\left(R\left(t\right)\right)=R\left(0\right)+\frac{1-\sigma }{q\left(\sigma \right)\sigma \Gamma \left(\sigma +1\right)N_{\sigma }\left(-\left(1/1-\sigma \right)V^{\sigma }\right)}\text{ST}\left[-aR+edS\right]. \end{array}$$

Now taking inverse ST on both sides of equation (52), we get

(57) $$\begin{array}{c} P\left(t\right)=P\left(0\right)+{\text{ST}}^{-1}\left[\frac{1-\sigma }{q\left(\sigma \right)\sigma \Gamma \left(\sigma +1\right)N_{\sigma }\left(-\left(1/1-\sigma \right)V^{\sigma }\right)}\text{ST}\left\{a\left(1-P\right)-bPS\right\}\right], \end{array}$$

(58) $$\begin{array}{c} L\left(t\right)=L\left(0\right)+{\text{ST}}^{-1}\left[\frac{1-\sigma }{q\left(\sigma \right)\sigma \Gamma \left(\sigma +1\right)N_{\sigma }\left(-\left(1/1-\sigma \right)V^{\sigma }\right)}\text{ST}\left\{-aL+bPL-cLS\right\}\right], \end{array}$$

(59) $$\begin{array}{c} S\left(t\right)=S\left(0\right)+{\text{ST}}^{-1}\left[\frac{1-\sigma }{q\left(\sigma \right)\sigma \Gamma \left(\sigma +1\right)N_{\sigma }\left(-\left(1/1-\sigma \right)V^{\sigma }\right)}\text{ST}\left\{-\left(a+d\right)S+cLS+fQ\right\}\right], \end{array}$$

(60) $$\begin{array}{c} Q\left(t\right)=Q\left(0\right)+{\text{ST}}^{-1}\left[\frac{1-\sigma }{q\left(\sigma \right)\sigma \Gamma \left(\sigma +1\right)N_{\sigma }\left(-\left(1/1-\sigma \right)V^{\sigma }\right)}\text{ST}\left\{-\left(a+f\right)Q+d\left(1-e\right)S\right\}\right], \end{array}$$

(61) $$\begin{array}{c} R\left(t\right)=R\left(0\right)+{\text{ST}}^{-1}\left[\frac{1-\sigma }{q\left(\sigma \right)\sigma \Gamma \left(\sigma +1\right)N_{\sigma }\left(-\left(1/1-\sigma \right)V^{\sigma }\right)}\text{ST}\left\{-aR+edS\right\}\right]. \end{array}$$

We next attain the following recursive formula.

(62) $$\begin{array}{c} P_{\left(n+1\right)}\left(t\right)=P_{n}\left(0\right)+{\text{ST}}^{-1}\left[\frac{1-\sigma }{q\left(\sigma \right)\sigma \Gamma \left(\sigma +1\right)N_{\sigma }\left(-\left(1/1-\sigma \right)V^{\sigma }\right)}\text{ST}\left\{a\left(1-P_{n}\right)-bP_{n}S_{n}\right\}\right], \end{array}$$

(63) $$\begin{array}{c} L_{\left(n+1\right)}\left(t\right)=L_{n}\left(0\right)+{\text{ST}}^{-1}\left[\frac{1-\sigma }{q\left(\sigma \right)\sigma \Gamma \left(\sigma +1\right)N_{\sigma }\left(-\left(1/1-\sigma \right)V^{\sigma }\right)}\text{ST}\left\{-aL_{n}+b{\text{P}}_{n}L_{n}-cL_{n}S_{n}\right\}\right], \end{array}$$

(64) $$\begin{array}{c} S_{n+1}\left(t\right)=S_{n}\left(0\right)+{\text{ST}}^{-1}\left[\frac{1-\sigma }{q\left(\sigma \right)\sigma \Gamma \left(\sigma +1\right)N_{\sigma }\left(-\left(1/1-\sigma \right)V^{\sigma }\right)}\text{ST}\left\{-\left(a+d\right)S_{n}+cL_{n}S_{n}+fQ_{n}\right\}\right], \end{array}$$

(65) $$\begin{array}{c} Q_{\left(n+1\right)}\left(t\right)=Q_{n}\left(0\right)+{\text{ST}}^{-1}\left[\frac{1-\sigma }{q\left(\sigma \right)\sigma \Gamma \left(\sigma +1\right)N_{\sigma }\left(-\left(1/1-\sigma \right)V^{\sigma }\right)}\text{ST}\left\{-\left(a+f\right)Q_{n}+d\left.\left(1-e\right)\right)S_{n}\right\}\right], \end{array}$$

(66) $$\begin{array}{c} R_{\left(n+1\right)}\left(t\right)=R_{n}\left(0\right)+{\text{ST}}^{-1}\left[\frac{1-\sigma }{q\left(\sigma \right)\sigma \Gamma \left(\sigma +1\right)N_{\sigma }\left(-\left(1/1-\sigma \right)V^{\sigma }\right)}\text{ST}\left\{-aR_{n}+edS_{n}\right\}\right]. \end{array}$$

And the solution of (62) is

(67) $$\begin{array}{c} P\left(t\right)=\underset{n⟶\infty }{\lim}P_{n}\left(t\right), \end{array}$$

(68) $$\begin{array}{c} L\left(t\right)=\underset{n⟶\infty }{\lim}L_{n}\left(t\right), \end{array}$$

(69) $$\begin{array}{c} S\left(t\right)=\underset{n⟶\infty }{\lim}S_{n}\left(t\right), \end{array}$$

(70) $$\begin{array}{c} Q\left(t\right)=\underset{n⟶\infty }{\lim}Q_{n}\left(t\right), \end{array}$$

(71) $$\begin{array}{c} R\left(t\right)=\underset{n⟶\infty }{\lim}R_{n}\left(t\right). \end{array}$$

**Theorem 3 .**

The article "Analysis and Simulation of Fractional Order Smoking Epidemic Model" was published in 2022. Journal: Comput Math Methods Med.

Let (*X*, |.|) be a Banach space and *H* a self-map of *X* satisfying

(72) $$\begin{array}{c} \left\|H_{x}-H_{r}\right\|\leq \theta \left\|X-H_{x}\right\|+\theta \left\|x-r\right\|, \end{array}$$

for all *x*, *r* ∈ *X*, and 0 ≤ *θ* < 1. Suppose that *H* is Picard *H*-stable. Suppose that system (62), we have

(73) $$\begin{array}{c} P_{n+1}\left(t\right)=P_{n}\left(0\right)+\text{S}{\text{T}}^{-1}\left\{\frac{1-\sigma }{q\left(\sigma \right)\sigma \Gamma \left(\sigma +1\right)N_{\sigma }\left(-\left(1/1-\sigma \right)V^{\sigma }\right)}\text{ST}\left[a\left(1-P_{n}\right)-bP_{n}S_{n}\right]\right\}, \end{array}$$

(74) $$\begin{array}{c} L_{n+1}\left(t\right)=L_{n}\left(0\right)+\text{S}{\text{T}}^{-1}\left\{\frac{1-\sigma }{q\left(\sigma \right)\sigma \Gamma \left(\sigma +1\right)N_{\sigma }\left(-\left(1/1-\sigma \right)V^{\sigma }\right)}\text{ST }\left[-aL_{n}+bP_{n}L_{n}-cL_{n}S_{n}\right]\right\}, \end{array}$$

(75) $$\begin{array}{c} S_{n+!}\left(t\right)=S_{n}\left(0\right)+\text{S}{\text{T}}^{-!}\left\{\frac{1-\sigma }{q\left(\sigma \right)\sigma \Gamma \left(\sigma +1\right)N_{\sigma }\left(-\left(1/1-\sigma \right)V^{\sigma }\right)}\text{ST}\left[-\left(a+d\right)S_{n}+cL_{n}S_{n}+fQ_{n}\right]\right\}, \end{array}$$

(76) $$\begin{array}{c} Q_{n+1}\left(t\right)=Q_{n}\left(0\right)+\text{S}{\text{T}}^{-1}\left\{\frac{1-\sigma }{q\left(\sigma \right)\sigma \Gamma \left(\sigma +1\right)N_{\sigma }\left(-\left(1/1-\sigma \right)V^{\sigma }\right)}\text{ ST}\left[-\left(a+f\right)Q_{n}+d\left(1-e\right)S_{n}\right]\right\}, \end{array}$$

(77) $$\begin{array}{c} R_{n+1}\left(t\right)=R_{n}\left(0\right)+\text{S}{\text{T}}^{-1}\left\{\frac{1-\sigma }{q\left(\sigma \right)\sigma \Gamma \left(\sigma +1\right)N_{\sigma }\left(-\left(1/1-\sigma \right)V^{\sigma }\right)}\text{ST}\left[-aR_{n}+edS_{n}\right]\right\}, \end{array}$$

where 1 − *σ*/*q*(*σ*)*σ*Γ(*σ* + 1)*N*_*σ*_(−1/1 − *σV*^*σ*^) is the fractional Lagrange multiplier.

The article "Analysis and Simulation of Fractional Order Smoking Epidemic Model" was published in 2022. Journal: Comput Math Methods Med.

**Theorem 4 .**

Define *K* be a self-map is given by

(78) $$\begin{array}{c} \text{K}\left[P_{\left(n+1\right)}\left(t\right)\right]=P_{n}\left(0\right)+{\text{ST}}^{-1}\left[\frac{1-\sigma }{q\left(\sigma \right)\sigma \Gamma \left(\sigma +1\right)N_{\sigma }\left(-\left(1/1-\sigma \right)V^{\sigma }\right)}\text{ST}\left\{a\left(1-P_{n}\right)-bP_{n}S_{n}\right\}\right], \end{array}$$

(79) $$\begin{array}{c} K\left[L_{\left(n+1\right)}\left(t\right)\right]=L_{n}\left(0\right)+{\text{ST}}^{-1}\left[\frac{1-\sigma }{q\left(\sigma \right)\sigma \Gamma \left(\sigma +1\right)N_{\sigma }\left(-\left(1/1-\sigma \right)V^{\sigma }\right)}\text{ST}\left\{-aL_{n}+bP_{n}L_{n}-cL_{n}S_{n}\right\}\right], \end{array}$$

(80) $$\begin{array}{c} K\left[S_{n+1}\left(t\right)\right]=S_{n}\left(0\right)+{\text{ST}}^{-1}\left[\frac{1-\sigma }{q\left(\sigma \right)\sigma \Gamma \left(\sigma +1\right)N_{\sigma }\left(-\left(1/1-\sigma \right)V^{\sigma }\right)}\text{ST}\left\{-\left(a+d\right)S_{n}+cL_{n}S_{n}+fQ_{n}\right\}\right], \end{array}$$

(81) $$\begin{array}{c} Q_{\left(n+1\right)}\left(t\right)=Q_{n}\left(0\right)+{\text{ST}}^{-1}\left[\frac{1-\sigma }{q\left(\sigma \right)\sigma \Gamma \left(\sigma +1\right)N_{\sigma }\left(-\left(1/1-\sigma \right)V^{\sigma }\right)}\text{ST}\left\{-\left(a+f\right)Q_{n}+d\left.\left(1-e\right)\right)S_{n}\right\}\right], \end{array}$$

(82) $$\begin{array}{c} R_{\left(n+1\right)}\left(t\right)=R_{n}\left(0\right)+{\text{ST}}^{-1}\left[\frac{1-\sigma }{q\left(\sigma \right)\sigma \Gamma \left(\sigma +1\right)N_{\sigma }\left(-\left(1/1-\sigma \right)V^{\sigma }\right)}\text{ST}\left\{-aR_{n}+edS_{n}\right\}\right], \end{array}$$

(83) $$\begin{array}{c} K\left[S_{n+1}\left(t\right)\right]=S_{n}\left(0\right)+{\text{ST}}^{-1}\left[\frac{1-\sigma }{q\left(\sigma \right)\sigma \Gamma \left(\sigma +1\right)N_{\sigma }\left(-\left(1/1-\sigma \right)V^{\sigma }\right)}\text{ST}\left\{-\left(a+d\right)S_{n}+cL_{n}S_{n}+fQ_{n}\right\}\right], \end{array}$$

(84) $$\begin{array}{c} K\left[Q_{\left(n+1\right)}\left(t\right)\right]=Q_{n}\left(0\right)+{\text{ST}}^{-1}\left[\frac{1-\sigma }{q\left(\sigma \right)\sigma \Gamma \left(\sigma +1\right)N_{\sigma }\left(-\left(1/1-\sigma \right)V^{\sigma }\right)}\text{ST}\left\{-\left(a+f\right)Q_{n}+d\left.\left(1-e\right)\right)S_{n}\right\}\right], \end{array}$$

(85) $$\begin{array}{c} K\left[R_{\left(n+1\right)}\left(t\right)\right]=R_{n}\left(0\right)+{\text{ST}}^{-1}\left[\frac{1-\sigma }{q\left(\sigma \right)\sigma \Gamma \left(\sigma +1\right)N_{\sigma }\left(-\left(1/1-\sigma \right)V^{\sigma }\right)}\text{ST}\left\{-aR_{n}+edS_{n}\right\}\right]. \end{array}$$

**Proof**

In first step, we will show that *K* is fixed point

(86) $$\begin{array}{c} \forall \left(m,n\right)\in N\times N, \end{array}$$

(87) $$\begin{array}{c} K\left(P_{n}\left(t\right)\right)-K\left(P_{m}\left(t\right)\right)=P_{n}\left(t\right)-P_{m}\left(t\right)+{\text{ST}}^{-1}\left[\frac{1-\sigma }{q\left(\sigma \right)\sigma \Gamma \left(\sigma +1\right)N_{\sigma }\left(-\left(1/1-\sigma \right)V^{\sigma }\right)}\text{ST}\left\{a\left(1-P_{n}\right)-bP_{n}S_{n}\right\}\right]-{\text{ST}}^{-1}\left[\frac{1-\sigma }{q\left(\sigma \right)\sigma \Gamma \left(\sigma +1\right)N_{\sigma }\left(-\left(1/1-\sigma \right)V^{\sigma }\right)}ST\left\{a\left(1-P_{m}\right)-bP_{m}S_{m}\right\}\right], \end{array}$$

(88) $$\begin{array}{c} K\left(L_{n}\left(t\right)\right)-K\left(L_{m}\left(t\right)\right)=L_{n}\left(t\right)-L_{m}\left(t\right)+{\text{ST}}^{-1}\left[\frac{1-\sigma }{q\left(\sigma \right)\sigma \Gamma \left(\sigma +1\right)N_{\sigma }\left(-\left(1/1-\sigma \right)V^{\sigma }\right)}\text{ST}\left\{-aL_{n}+bP_{n}L_{n}-cL_{n}S_{n}\right\}\right]-{\text{ST}}^{-1}\left[\frac{1-\sigma }{q\left(\sigma \right)\sigma \Gamma \left(\sigma +1\right)N_{\sigma }\left(-\left(1/1-\sigma \right)V^{\sigma }\right)}\text{ST}\left\{-aL_{m}+bP_{m}L_{m}-cL_{m}S_{m}\right\}\right], \end{array}$$

(89) $$\begin{array}{c} K\left(S_{n}\left(t\right)\right)-K\left(S_{m}\left(t\right)\right)=S_{n}\left(t\right)-S_{m}\left(t\right)+{\text{ST}}^{-1}\left[\frac{1-\sigma }{q\left(\sigma \right)\sigma \Gamma \left(\sigma +1\right)N_{\sigma }\left(-\left(1/1-\sigma \right)V^{\sigma }\right)}\text{ST}\left\{-\left(a+d\right)S_{n}+cL_{n}S_{n}+fQ_{n}\right\}\right]-{\text{ST}}^{-1}\left[\frac{1-\sigma }{q\left(\sigma \right)\sigma \Gamma \left(\sigma +1\right)N_{\sigma }\left(-\left(1/1-\sigma \right)V^{\sigma }\right)}\text{ST}\left\{-\left(a+d\right)S_{m}+cL_{m}S_{m}+fQ_{m}\right\}\right], \end{array}$$

(90) $$\begin{array}{c} K\left(Q_{n}\left(t\right)\right)-K\left(Q_{m}\left(t\right)\right)=Q_{n}\left(t\right)-Q_{m}\left(t\right)+{\text{ST}}^{-1}\left[\frac{1-\sigma }{q\left(\sigma \right)\sigma \Gamma \left(\sigma +1\right)N_{\sigma }\left(-\left(1/1-\sigma \right)V^{\sigma }\right)}ST\left\{-\left(a+f\right)Q_{n}+d\left.\left(1-e\right)\right)S_{n}\right\}\right]-{\text{ST}}^{-1}\left[\frac{1-\sigma }{q\left(\sigma \right)\sigma \Gamma \left(\sigma +1\right)N_{\sigma }\left(-\left(1/1-\sigma \right)V^{\sigma }\right)}\text{ST}\left\{-\left(a+f\right)Q_{m}+d\left.\left(1-e\right)\right)S_{m}\right\}\right], \end{array}$$

(91) $$\begin{array}{c} K\left(R_{n}\left(t\right)\right)-K\left(R\left(t\right)\right)=R_{n}\left(t\right)-R_{m}\left(t\right)+{\text{ST}}^{-1}\left[\frac{1-\sigma }{q\left(\sigma \right)\sigma \Gamma \left(\sigma +1\right)N_{\sigma }\left(-\left(1/1-\sigma \right)V^{\sigma }\right)}\text{ST}\left\{-aR_{n}+edS_{n}\right\}\right]-{\text{ST}}^{-1}\left[\frac{1-\sigma }{q\left(\sigma \right)\sigma \Gamma \left(\sigma +1\right)N_{\sigma }\left(-\left(1/1-\sigma \right)V^{\sigma }\right)}\text{ST}\left\{-aR_{m}+edS_{m}\right\}\right]. \end{array}$$

Applying the properties of the norm and also using the triangular inequality, we obtain

(92) $$\begin{array}{c} \left\|K\left(P_{n}\left(t\right)\right)-K\left(P_{m}\left(t\right)\right)\right\|\leq \left\|P_{n}\left(t\right)-P_{m}\left(t\right)\right\|\text{ S}{\text{T}}^{-1}\left[\frac{1-\sigma }{q\left(\sigma \right)\sigma \Gamma \left(\sigma +1\right)N_{\sigma }\left(-\left(1/1-\sigma \right)V^{\sigma }\right)}\text{ST}\left\{\left\|a\left(1-\left(P_{n}-P_{m}\right)\right)\right\|\right.+\left\|-b\left(P_{n}S_{n}-P_{m}S_{m}\right)\right\|\right], \end{array}$$

(93) $$\begin{array}{c} \left\|K\left(L_{n}\left(t\right)\right)-K\left(L_{m}\left(t\right)\right)\right\|\leq \left\|L_{n}\left(t\right)-L_{m}\left(t\right)\right\|+{\text{ST}}^{-1}\left[\frac{1-\sigma }{q\left(\sigma \right)\sigma \Gamma \left(\sigma +1\right)N_{\sigma }\left(-\left(1/1-\sigma \right)V^{\sigma }\right)}\text{ST}\left\{-\left\|a\left(L_{n}-L_{m}\right)\right\|+\left\|b\left(P_{n}L_{n}-P_{m}L_{m}\right)\right\|+\left\|-c\left(L_{n}S_{n}-L_{m}S_{m}\right)\right\|\right\}\right], \end{array}$$

(94) $$\begin{array}{c} \left\|K\left(S_{n}\left(t\right)\right)-K\left(S_{m}\left(t\right)\right)\right\|\leq \left\|S_{n}\left(t\right)-S_{m}\left(t\right)\right\|+{\text{ST}}^{-1}\left[\frac{1-\sigma }{q\left(\sigma \right)\sigma \Gamma \left(\sigma +1\right)N_{\sigma }\left(-\left(1/1-\sigma \right)V^{\sigma }\right)}\text{ST}\left\{-\left\|\left(a+d\right)\left(S_{n}-S_{m}\right)\right\|+\left\|c\left(L_{n}S_{n}-L_{m}S_{m}\right)\right\|+\left\|f\left(Q_{n}-Q_{m}\right)\right\|\right\}\right], \end{array}$$

(95) $$\begin{array}{c} \left\|K\left(Q_{n}\left(t\right)\right)-K\left(Q_{m}\left(t\right)\right)\right\|\leq \left\|Q_{n}\left(t\right)-Q_{m}\left(t\right)\right\|+{\text{ST}}^{-1}\left[\frac{1-\sigma }{q\left(\sigma \right)\sigma \Gamma \left(\sigma +1\right)N_{\sigma }\left(-\left(1/1-\sigma \right)V^{\sigma }\right)}\text{ST}\left\{-\left\|\left(a+f\right)\left(Q_{n}-Q_{m}\right)\right\|+\left\|d\left(1-e\right)\left(S_{n}-S_{m}\right)\right\|\right\}\right], \end{array}$$

(96) $$\begin{array}{c} \left\|K\left(R_{n}\left(t\right)\right)-K\left(R_{m}\left(t\right)\right)\right\|\leq \left\|R_{n}\left(t\right)-R_{m}\left(t\right)\right\|+{ST}^{-1}\left[\frac{1-\sigma }{q\left(\sigma \right)\sigma \Gamma \left(\sigma +1\right)N_{\sigma }\left(-\left(1/1-\sigma \right)V^{\sigma }\right)}\text{ST}\left\{\left\|-a\left(R_{n}-R_{m}\right)\right\|+\left\|ed\left(S_{n}-S_{m}\right)\right\|\right\}\right]. \end{array}$$

*K* fulfills the conditions associated with Theorem 6, when

(97) $$\begin{array}{c} \theta =\left(0,0,0,0,0\right),\theta \left\{\begin{array}{c} \left\|{\text{P}}_{\text{n}}\left(\text{t}\right)-{\text{P}}_{\text{m}}\left(\text{t}\right)\right\|\times \left\|-{\text{P}}_{\text{n}}\left(\text{t}\right)-{\text{P}}_{\text{m}}\left(\text{t}\right)\right\|+\text{a}\left\|\left(1-\left({\text{P}}_{\text{n}}-{\text{P}}_{\text{m}}\right)\right)\right\|-\text{b}\left\|\left({\text{P}}_{\text{n}}{\text{S}}_{\text{n}}-{\text{P}}_{\text{m}}{\text{S}}_{\text{m}}\right)\right\|,\\ \times \left\|{\text{L}}_{\text{n}}\left(\text{t}\right)-{\text{L}}_{\text{m}}\left(\text{t}\right)\right\|\times \left\|-{\text{L}}_{\text{n}}\left(\text{t}\right)-{\text{L}}_{\text{m}}\left(\text{t}\right)\right\|-\text{a}\left\|{\text{L}}_{\text{n}}\left(\text{t}\right)-{\text{L}}_{\text{m}}\left(\text{t}\right)\right\|+\text{b}\left\|\left({\text{P}}_{\text{n}}{\text{L}}_{\text{n}}-{\text{P}}_{\text{m}}{\text{L}}_{\text{m}}\right)\right\|-\text{c}\left\|\left({\text{L}}_{\text{n}}{\text{S}}_{\text{n}}-{\text{L}}_{\text{m}}{\text{S}}_{\text{m}}\right)\right\|,\\ \times \left\|{\text{S}}_{\text{n}}\left(\text{t}\right)-{\text{S}}_{\text{m}}\left(\text{t}\right)\right\|\times \left\|-{\text{S}}_{\text{n}}\left(\text{t}\right)-{\text{S}}_{\text{m}}\left(\text{t}\right)\right\|-\left(\text{a}+\text{d}\right)\left\|{\text{P}}_{\text{n}}-{\text{P}}_{\text{m}}\right\|+\text{c}\left\|\left({\text{L}}_{\text{n}}{\text{S}}_{\text{n}}-{\text{L}}_{\text{m}}{\text{S}}_{\text{m}}\right)\right\|+\text{f}\left\|\left({\text{Q}}_{\text{n}}-{\text{Q}}_{\text{m}}\right)\right\|,\\ \times \left\|{\text{Q}}_{\text{n}}\left(\text{t}\right)-{\text{Q}}_{\text{m}}\left(\text{t}\right)\right\|\times \left\|-{\text{Q}}_{\text{n}}\left(\text{t}\right)-{\text{Q}}_{\text{m}}\left(\text{t}\right)\right\|-\left(\text{a}+\text{f}\right)\left\|{\text{Q}}_{\text{n}}-{\text{Q}}_{\text{m}}\right\|+\text{d}\left(1-\text{e}\right)\left\|\text{d}\left(1-\text{e}\right)\left({\text{S}}_{\text{n}}-{\text{S}}_{\text{m}}\right)\right\|,\\ \times \left\|{\text{R}}_{\text{n}}\left(\text{t}\right)-{\text{R}}_{\text{m}}\left(\text{t}\right)\right\|\times \left\|-{\text{R}}_{\text{n}}\left(\text{t}\right)-{\text{R}}_{\text{m}}\left(\text{t}\right)\right\|-\text{a}\left\|{\text{R}}_{\text{n}}-{\text{R}}_{\text{m}}\right\|+\text{ed}\left\|\left({\text{S}}_{\text{n}}-{\text{S}}_{\text{m}}\right)\right\|. \end{array}\right. \end{array}$$

And we add that *K* is Picard *K*-stable.

The article "Analysis and Simulation of Fractional Order Smoking Epidemic Model" was published in 2022. Journal: Comput Math Methods Med.

**Theorem 5 .**

Prove that system (27) has special solution is unique.

**Proof**

Let *H* be the Hilbert space defined as *H* = *L*^2^((*p*, *q*) × (0, *T*)) where

(98) $$\begin{array}{c} h:\left(p,q\right)\times \left(0,T\right)⟶\mathbb{R},\iint ghdgdh<\infty . \end{array}$$

So, the following operators are considered

(99) $$\begin{array}{c} \theta \left(0,0,0,0,0\right),\theta =\left\{\begin{array}{c} \text{a}\left(1-\text{p}\right)-\text{bps},\\ -aL+bPL-cLS,\\ -\left(a+d\right)S+cLS+fQ,\\ -\left(a+f\right)Q+d\left(1-e\right)S,\\ -aR+edS. \end{array}\right. \end{array}$$

We establish the inner product of

(100) $$\begin{array}{c} P\left(\left(P_{11}-P_{12},L_{21}-L_{22},S_{31}-S_{32},Q_{41}-Q_{42},R_{51}-R_{52}\right),\left(V_{1},V_{2},V_{3},V_{4},V_{5}\right)\right). \end{array}$$

where (*S*_11_ − *S*_12_, *I*_21_ − *I*_22_, *A*_31_ − *A*_32_, *T*_41_ − *T*_42_, *R*_51_ − *R*_52_) are the special solutions of the system. By using the inner function and the norm, we have

(101) $$\begin{array}{c} \left\{a-a\left(P_{11}-P_{12}\right)-b\left(P_{11}-P_{12}\right)\left(S_{31}-S_{32}\right)\right\}\leq a\left\|V_{1}\right\|+a\left\|P_{11}-P_{12}\right\|+b\left\|P_{11}-P_{12}\right\|\times \left\|S_{31}-S_{32}\right\|\left\|V_{1}\right\|, \end{array}$$

(102) $$\begin{array}{c} \left\{-\text{a}\left({\text{L}}_{21}-{\text{L}}_{22}\right)+\text{b}\left({\text{P}}_{11}-{\text{P}}_{12}\right)\left({\text{L}}_{21}-{\text{L}}_{22}\right)-\text{c}\left({\text{L}}_{21}-{\text{L}}_{22}\right)\left({\text{S}}_{31}-{\text{S}}_{32}\right)\right\}\leq \text{a}\left\|{\text{L}}_{21}-{\text{L}}_{22}\right\|\left\|{\text{V}}_{2}\right\|+\text{b}\left\|{\text{P}}_{11}-{\text{P}}_{12}\right\|\left\|{\text{L}}_{21}-{\text{L}}_{22}\right\|\left\|{\text{V}}_{2}\right\|+\text{c}\left\|{\text{L}}_{21}-{\text{L}}_{22}\right\|\left\|{\text{S}}_{31}-{\text{S}}_{32}\right\|\left\|{\text{V}}_{2}\right\|, \end{array}$$

(103) $$\begin{array}{c} \left\{-\left(\text{a}+\text{d}\right)\left({\text{S}}_{31}-{\text{S}}_{32}\right)+\text{c}\left({\text{L}}_{21}-{\text{L}}_{22}\right)\left({\text{S}}_{31}-{\text{S}}_{32}\right)+\text{f}\left({\text{Q}}_{41}-{\text{Q}}_{42}\right)\right\}\leq \left(\text{a}+\text{d}\right)\left\|{\text{S}}_{31}-{\text{S}}_{32}\right\|\left\|{\text{V}}_{3}\right\|+\text{c}\left\|{\text{L}}_{21}-{\text{L}}_{22}\right\|\left\|{\text{S}}_{31}-{\text{S}}_{32}\right\|\left\|{\text{V}}_{3}\right\|+\text{f}\left\|{\text{Q}}_{31}-{\text{Q}}_{32}\right\|\left\|{\text{V}}_{3}\right\|, \end{array}$$

(104) $$\begin{array}{c} \left\{-\left(\text{a}+\text{f}\right)\left({\text{Q}}_{41}-{\text{Q}}_{42}\right)+\text{d}\left(1-\text{e}\right)\left({\text{S}}_{31}-{\text{S}}_{32}\right)\right\}\leq \left(\text{a}+\text{f}\right)\left\|{\text{Q}}_{31}-{\text{Q}}_{32}\right\|\left\|{\text{V}}_{4}\right\|+\text{d}\left(1-\text{e}\right)\left\|{\text{S}}_{31}-{\text{S}}_{32}\right\|\left\|{\text{V}}_{4}\right\|, \end{array}$$

(105) $$\begin{array}{c} \left\{-\text{a}\left({\text{R}}_{51}-{\text{R}}_{52}\right)+\text{ed}\left({\text{S}}_{31}-{\text{S}}_{32}\right)\right\}\leq \text{a}\left\|{\text{R}}_{31}-{\text{R}}_{32}\right\|\left\|{\text{V}}_{5}\right\|+\text{ed}\left\|{\text{S}}_{31}-{\text{S}}_{32}\right\|\left\|{\text{V}}_{5}\right\|. \end{array}$$

Due to large number of *e*_1_, *e*_2_,  *e*_3_,  *e*_4_, and  *e*_5_, both solutions converge to the exact solution. Applying the topological idea, we have the very small positive five parameters (*χ*_*e*_1__,  *χ*_*e*_2__,  *χ*_*e*_3__, *χ*_*e*_4__, and *χ*_*e*_5__).

(106) $$\begin{array}{c} \left\|P-P_{11}\right\|,\left\|P-P_{12}\right\|\leq \frac{\chi_{e_{1}}}{\varpi }, \end{array}$$

(107) $$\begin{array}{c} \left\|L-L_{21}\right\|,\left\|L-L_{22}\right\|\leq \frac{\chi_{e_{2}}}{\varsigma }, \end{array}$$

(108) $$\begin{array}{c} \left\|S-S_{31}\right\|,\left\|S-S_{32}\right\|\leq \frac{\chi_{e_{3}}}{\upsilon }, \end{array}$$

(109) $$\begin{array}{c} \left\|Q-Q_{41}\right\|,\left\|Q-Q_{42}\right\|\leq \frac{\chi_{e_{4}}}{\kappa }, \end{array}$$

(110) $$\begin{array}{c} \left\|R-R_{51}\right\|,\left\|R-R_{52}\right\|\leq \frac{\chi_{e_{5}}}{\varrho }, \end{array}$$

(111) $$\begin{array}{c} \varpi =5\left(a+a\left\|P_{11}-P_{12}\right\|+b\left\|P_{11}-P_{12}\right\|\left\|S_{31}-S_{32}\right\|\right)\left\|V_{1}\right\|, \end{array}$$

(112) $$\begin{array}{c} \varsigma =5\left(a\left\|L_{21}-L_{22}\right\|+b\left\|P_{11}-P_{12}\right\|\left\|L_{21}-L_{22}\right\|+c\left\|L_{21}-L_{22}\right\|\left\|S_{31}-S_{32}\right\|\right)\left\|V_{2}\right\|, \end{array}$$

(113) $$\begin{array}{c} \upsilon =5\left(\left(a+d\right)\left\|S_{31}-S_{32}\right\|+c\left\|L_{21}-L_{22}\right\|\left\|S_{31}-S_{32}\right\|+f\left\|Q_{31}-Q_{32}\right\|\right)\left\|V_{3}\right\|, \end{array}$$

(114) $$\begin{array}{c} \kappa =5\left(\left(a+f\right)\left\|Q_{31}-Q_{32}\right\|+d\left(1-e\right)\left\|S_{31}-S_{32}\right\|\right)\left\|V_{4}\right\|, \end{array}$$

(115) $$\begin{array}{c} \varrho =5\left(a\left\|R_{31}-R_{32}\right\|+ed\left\|S_{31}-S_{32}\right\|\right)\left\|V_{5}\right\|. \end{array}$$

But, it is obvious that

(116) $$\begin{array}{c} \left(a+a\left\|P_{11}-P_{12}\right\|+b\left\|P_{11}-P_{12}\right\|\left\|S_{31}-S_{32}\right\|\right)\neq 0, \end{array}$$

(117) $$\begin{array}{c} \left(a\left\|L_{21}-L_{22}\right\|+b\left\|P_{11}-P_{12}\right\|\left\|L_{21}-L_{22}\right\|+c\left\|L_{21}-L_{22}\right\|\left\|S_{31}-S_{32}\right\|\right)\neq 0, \end{array}$$

(118) $$\begin{array}{c} \left(\left(a+d\right)\left\|S_{31}-S_{32}\right\|+c\left\|L_{21}-L_{22}\right\|\left\|S_{31}-S_{32}\right\|+f\left\|Q_{31}-Q_{32}\right\|\right)\neq 0, \end{array}$$

(119) $$\begin{array}{c} \left(\left(a+f\right)\left\|Q_{31}-Q_{32}\right\|+d\left(1-e\right)\left\|S_{31}-S_{32}\right\|\right)\neq 0, \end{array}$$

(120) $$\begin{array}{c} \left(a\left\|R_{31}-R_{32}\right\|+ed\left\|S_{31}-S_{32}\right\|\right)\neq 0, \end{array}$$

where ‖*V*_1_‖, ‖*V*_2_‖, ‖*V*_3_‖, ‖*V*_4_‖, ‖*V*_5_‖ ≠ 0.

The article "Analysis and Simulation of Fractional Order Smoking Epidemic Model" was published in 2022. Journal: Comput Math Methods Med.

Therefore, we have

(121) $$\begin{array}{c} \left\|P_{11}-P_{12}\right\|=0, \end{array}$$

(122) $$\begin{array}{c} \left\|L_{21}-L_{22}\right\|=0, \end{array}$$

(123) $$\begin{array}{c} \left\|S_{31}-S_{32}\right\|=0, \end{array}$$

(124) $$\begin{array}{c} \left\|Q_{41}-Q_{42}\right\|=0, \end{array}$$

(125) $$\begin{array}{c} \left\|R_{51}-R_{52}\right\|=0. \end{array}$$

Which yields that

(126) $$\begin{array}{c} P_{11}=P_{12}, \end{array}$$

(127) $$\begin{array}{c} L_{21}=L_{22}, \end{array}$$

(128) $$\begin{array}{c} S_{31}=S_{32}, \end{array}$$

(129) $$\begin{array}{c} Q_{41}=Q_{42}, \end{array}$$

(130) $$\begin{array}{c} R_{51}=R_{52}. \end{array}$$

This completes the proof of uniqueness.

## 6. New Numerical Scheme

We define the AT proposed scheme for fractional derivative model (37) for the smoking epidemic. For this purpose, we suppose that we obtain the following results for system (37)

(131) $$\begin{array}{c} P\left(t\right)-P\left(0\right)=\frac{\left(1-\sigma \right)}{\text{ABC}\left(\sigma \right)}\left\{\text{a}-aP\left(t\right)-bP\left(t\right)S\left(t\right)\right\}+\frac{\sigma }{\Gamma \left(\sigma \right)\times \text{ABC}\left(\sigma \right)}\int_{0}^{t}\left\{\text{a}-aP\left(\tau \right)-bP\left(\tau \right)S\left(\tau \right)\right\}{\left(t-\tau \right)}^{\sigma -1}d\tau , \end{array}$$

(132) $$\begin{array}{c} L\left(t\right)-L\left(0\right)=\frac{\left(1-\sigma \right)}{\text{ABC}\left(\sigma \right)}\left\{-aL\left(t\right)+bP\left(t\right)L\left(t\right)-cL\left(t\right)S\left(t\right)\right\}+\frac{\sigma }{\Gamma \left(\sigma \right)\times \text{ABC}\left(\sigma \right)}\int_{0}^{t}\left\{-aL\left(\tau \right)+bP\left(t\right)L\left(\tau \right)-cL\left(\tau \right)S\left(\tau \right)\right\}{\left(t-\tau \right)}^{\sigma -1}d\tau , \end{array}$$

(133) $$\begin{array}{c} S\left(t\right)-S\left(0\right)=\frac{\left(1-\sigma \right)}{ABC\left(\sigma \right)}\left\{-\left(a+d\right)S\left(t\right)+cL\left(t\right)S\left(t\right)+fQ\left(t\right)\right\}+\frac{\sigma }{\Gamma \left(\sigma \right)\times ABC\left(\sigma \right)}\int_{0}^{t}\left\{-\left(a+d\right)S\left(\tau \right)+cL\left(t\right)S\left(\tau \right)+fQ\left(\tau \right)\right\}{\left(t-\tau \right)}^{\sigma -1}d\tau , \end{array}$$

(134) $$\begin{array}{c} Q\left(t\right)-Q\left(0\right)=\frac{\left(1-\sigma \right)}{\text{ABC}\left(\sigma \right)}\left\{-\left(a+f\right)Q\left(t\right)+d\left(1-e\right)S\left(t\right)\right\}+\frac{\sigma }{\Gamma \left(\sigma \right)\times \text{ABC}\left(\sigma \right)}\int_{0}^{t}\left\{-\left(a+f\right)Q\left(\tau \right)+d\left(1-e\right)S\left(\tau \right)\right\}{\left(t-\tau \right)}^{\sigma -1}d\tau , \end{array}$$

(135) $$\begin{array}{c} R\left(t\right)-R\left(0\right)=\frac{\left(1-\sigma \right)}{\text{ABC}\left(\sigma \right)}\left\{-aR\left(t\right)+edS\left(t\right)\right\}+\frac{\sigma }{\Gamma \left(\sigma \right)\times \text{ABC}\left(\sigma \right)}\int_{0}^{t}\left\{-aR\left(\tau \right)+edS\left(\tau \right)\right\}{\left(t-\tau \right)}^{\sigma -1}d\tau . \end{array}$$

At a given point *t*_*n*+1_, *n* = 0, 1, 2, 3, ⋯, the above equation is reformulated as

(136) $$\begin{array}{c} P\left(t\right)-P\left(0\right)=\frac{\left(1-\sigma \right)}{\text{ABC}\left(\sigma \right)}\left\{\text{a}-aP\left(t_{n}\right)-bP\left(t_{n}\right)S\left(t_{n}\right)\right\}+\frac{\sigma }{\Gamma \left(\sigma \right)\times \text{ABC}\left(\sigma \right)}\int_{0}^{t}\left\{\text{a}-aP\left(\tau \right)-bP\left(\tau \right)S\left(\tau \right)\right\}{\left(t-\tau \right)}^{\sigma -1}d\tau , \end{array}$$

(137) $$\begin{array}{c} L\left(t\right)-L\left(0\right)=\frac{\left(1-\sigma \right)}{\text{ABC}\left(\sigma \right)}\left\{-aL\left(t_{n}\right)+bP\left(t_{n}\right)L\left(t_{n}\right)-cL\left(t_{n}\right)S\left(t_{n}\right)\right\}+\frac{\sigma }{\Gamma \left(\sigma \right)\times \text{ABC}\left(\sigma \right)}\int_{0}^{t}\left\{-aL\left(\tau \right)+bP\left(\tau \right)L\left(\tau \right)-cL\left(\tau \right)S\left(\tau \right)\right\}{\left(t-\tau \right)}^{\sigma -1}d\tau , \end{array}$$

(138) $$\begin{array}{c} S\left(t\right)-S\left(0\right)=\frac{\left(1-\sigma \right)}{\text{ABC}\left(\sigma \right)}\left\{-\left(a+d\right)S\left(t_{n}\right)+cL\left(t_{n}\right)S\left(t_{n}\right)+fQ\left(t_{n}\right)\right\}+\frac{\sigma }{\Gamma \left(\sigma \right)\times \text{ABC}\left(\sigma \right)}\int_{0}^{t}\left\{-\left(a+d\right)S\left(\tau \right)+cL\left(\tau \right)S\left(\tau \right)+fQ\left(\tau \right)\right\}{\left(t-\tau \right)}^{\sigma -1}d\tau , \end{array}$$

(139) $$\begin{array}{c} Q\left(t\right)-Q\left(0\right)=\frac{\left(1-\sigma \right)}{\text{ABC}\left(\sigma \right)}\left\{-\left(a+f\right)Q\left(t_{n}\right)+d\left(1-e\right)S\left(t_{n}\right)\right\}+\frac{\sigma }{\Gamma \left(\sigma \right)\times \text{ABC}\left(\sigma \right)}\int_{0}^{t}\left\{-\left(a+f\right)Q\left(\tau \right)+d\left(1-e\right)S\left(\tau \right)\right\}{\left(t-\tau \right)}^{\sigma -1}d\tau , \end{array}$$

(140) $$\begin{array}{c} R\left(t\right)-R\left(0\right)=\frac{\left(1-\sigma \right)}{\text{ABC}\left(\sigma \right)}\left\{-aR\left(t_{n}\right)+edS\left(t_{n}\right)\right\}+\frac{\sigma }{\Gamma \left(\sigma \right)\times \text{ABC}\left(\sigma \right)}\int_{0}^{t}\left\{-aR\left(\tau \right)+edS\left(\tau \right)\right\}{\left(t-\tau \right)}^{\sigma -1}d\tau . \end{array}$$

Also, we have

(141) $$\begin{array}{c} P\left(t_{n+1}\right)-P\left(0\right)=\frac{\left(1-\sigma \right)}{\text{ABC}\left(\sigma \right)}\left\{\text{a}-aP\left(t_{n}\right)-bP\left(t_{n}\right)S\left(t_{n}\right)\right\}+\frac{\sigma }{\Gamma \left(\sigma \right)\times \text{ABC}\left(\sigma \right)}\overset{n}{\underset{j=0}{\sum }}\int_{t_{j}}^{t_{j+1}}\left\{\text{a}-aP\left(\tau \right)-bP\left(\tau \right)S\left(\tau \right)\right\}{\left(t_{n+1}-\tau \right)}^{\sigma -1}d\tau , \end{array}$$

(142) $$\begin{array}{c} L\left(t_{n+1}\right)-L\left(0\right)=\frac{\left(1-\sigma \right)}{\text{ABC}\left(\sigma \right)}\left\{-aL\left(t_{n}\right)+bP\left(t_{n}\right)L\left(t_{n}\right)-cL\left(t_{n}\right)S\left(t_{n}\right)-cL\left(\tau \right)S\left(\tau \right)\right\}+\frac{\sigma }{\Gamma \left(\sigma \right)\times \text{ABC}\left(\sigma \right)}\overset{n}{\underset{j=0}{\sum }}\int_{t_{j}}^{t_{j+1}}\left\{-\text{a}L\left(\tau \right)+bP\left(\tau \right)L\left(\tau \right)-cL\left(\tau \right)S\left(\tau \right)\right\}{\left(t_{n+1}-\tau \right)}^{\sigma -1}d\tau , \end{array}$$

(143) $$\begin{array}{c} S\left(t_{n+1}\right)-S\left(0\right)=\frac{\left(1-\sigma \right)}{\text{ABC}\left(\sigma \right)}\left\{-\left(a+d\right)S\left(t_{n}\right)+cL\left(t_{n}\right)S\left(t_{n}\right)+fQ\left(t_{n}\right)\right\}+\frac{\sigma }{\Gamma \left(\sigma \right)\times \text{ABC}\left(\sigma \right)}\overset{n}{\underset{j=0}{\sum }}\int_{t_{j}}^{t_{j+1}}\left\{-\left(\text{a}+\text{d}\right)\text{S}\left(\tau \right)+cL\left(\tau \right)S\left(\tau \right)+fQ\left(\tau \right)\right\}{\left(t_{n+1}-\tau \right)}^{\sigma -1}d\tau , \end{array}$$

(144) $$\begin{array}{c} Q\left(t_{n+1}\right)-Q\left(0\right)=\frac{\left(1-\sigma \right)}{\text{ABC}\left(\sigma \right)}\left\{-\left(a+f\right)Q\left(t_{n}\right)+d\left(1-e\right)S\left(t_{n}\right)\right\}+\frac{\sigma }{\Gamma \left(\sigma \right)\times \text{ABC}\left(\sigma \right)}\overset{n}{\underset{j=0}{\sum }}\int_{t_{j}}^{t_{j+1}}\left\{-\left(\text{a}+\text{f}\right)\text{Q}\left(\tau \right)+d\left(1-e\right)S\left(\tau \right)\right\}{\left(t_{n+1}-\tau \right)}^{\sigma -1}d\tau , \end{array}$$

(145) $$\begin{array}{c} R\left(t_{n+1}\right)-R\left(0\right)=\frac{\left(1-\sigma \right)}{\text{ABC}\left(\sigma \right)}\left\{-aR\left(t_{n}\right)+edS\left(t_{n}\right)\right\}+\frac{\sigma }{\Gamma \left(\sigma \right)\times \text{ABC}\left(\sigma \right)}\overset{n}{\underset{j=0}{\sum }}\int_{{\text{t}}_{j}}^{t_{j+1}}\left\{-aR\left(\tau \right)+edS\left(\tau \right)\right\}{\left(t_{n+1}-\tau \right)}^{\sigma -1}d\tau . \end{array}$$

By using equation (133), we have

(146) $$\begin{array}{c} \begin{array}{c} P_{n+1}=P_{0}+\frac{\left(1-\sigma \right)}{ABC\left(\sigma \right)}\left\{\text{a}-aP\left(t_{n}\right)-bP\left(t_{n}\right)S\left(t_{n}\right)\right\}+\frac{\sigma }{\Gamma \left(\sigma \right)\times ABC\left(\sigma \right)}\\ \cdot \overset{n}{\underset{j=0}{\sum }}\left(\frac{\left\{\text{a}-aP_{j}-bP_{j}S_{j}\right\}}{h}\right.\times \int_{t_{j}}^{t_{j+1}}\left(\tau -t_{j-1}\right){\left(t_{n+1}-\tau \right)}^{\sigma -1}d\tau \\ -\frac{\left\{\text{a}-aP_{j-1}-bP_{j-1}S_{j-1}\right\}}{h}\times \left.\int_{t_{j}}^{t_{j+1}}\left(\tau -t_{j}\right){\left(t_{n+1}-\tau \right)}^{\sigma -1}d\tau \right), \end{array} \end{array}$$

(147) $$\begin{array}{c} \begin{array}{c} L_{n+1}=L_{0}+\frac{\left(1-\sigma \right)}{\text{ABC}\left(\sigma \right)}\left\{-aL\left(t_{n}\right)+bP\left(t_{n}\right)L\left(t_{n}\right)-cL\left(t_{n}\right)S\left(t_{n}\right)\right\}\\ +\frac{\sigma }{\Gamma \left(\sigma \right)\times \text{ABC}\left(\sigma \right)}\overset{n}{\underset{j=0}{\sum }}\left(\frac{\left\{-aL_{j}+bP_{j}L_{j}-cL_{j}S_{j}\right\}}{h}\right.\\ \times \int_{t_{j}}^{t_{j+1}}\left(\tau -t_{j-1}\right){\left(t_{n+1}-\tau \right)}^{\sigma -1}d\tau \\ \left.-\frac{\left\{-aL_{j-1}+bP_{j-1}L_{j-1}-cL_{j-1}S_{j-1}\right\}}{h}\times \int_{t_{j}}^{t_{j+1}}\left(\tau -t_{j}\right){\left(t_{n+1}-\tau \right)}^{\sigma -1}d\tau \right), \end{array} \end{array}$$

(148) $$\begin{array}{c} \begin{array}{c} S_{n+1}=S_{0}+\frac{\left(1-\sigma \right)}{\text{ABC}\left(\sigma \right)}\left\{-\left(a+d\right)S\left(t_{n}\right)+cL\left(t_{n}\right)S\left(t_{n}\right)+fQ\left(t_{n}\right)\right\}\\ +\frac{\sigma }{\Gamma \left(\sigma \right)\times \text{ABC}\left(\sigma \right)}\overset{n}{\underset{j=0}{\sum }}\left(\frac{\left\{-\left(a+d\right)S_{j}+cL_{j}S_{j}+fQ_{j}\right\}}{h}\right.\\ \times \int_{t_{j}}^{t_{j+1}}\left(\tau -t_{j-1}\right){\left(t_{n+1}-\tau \right)}^{\sigma -1}d\tau \\ \left.-\frac{\left\{-\left(a+d\right)S_{j-1}+cL_{j-1}S_{j-1}+fQ_{j-1}\right\}}{h}\times \int_{t_{j}}^{t_{j+1}}\left(\tau -t_{j}\right){\left(t_{n+1}-\tau \right)}^{\sigma -1}d\tau \right), \end{array} \end{array}$$

(149) $$\begin{array}{c} \begin{array}{c} Q_{n+1}=Q_{0}+\frac{\left(1-\sigma \right)}{\text{ABC}\left(\sigma \right)}\left\{-\left(a+f\right)Q\left(t_{n}\right)+d\left(1-e\right)S\left(t_{n}\right)\right\}\\ +\frac{\sigma }{\Gamma \left(\sigma \right)\times \text{ABC}\left(\sigma \right)}\overset{n}{\underset{j=0}{\sum }}\left(\frac{\left\{-\left(a+f\right)Q_{j}+d\left(1-e\right)S_{j}\right\}}{h}\right.\\ \times \int_{t_{j}}^{t_{j+1}}{\left(\tau -t_{j-1}\right)\left(t_{n+1}-\tau \right)}^{\sigma -1}d\tau \\ \left.-\frac{\left\{-\left(a+f\right)Q_{j-1}+d\left(1-e\right)S_{j-1}\right\}}{h}\times \int_{t_{j}}^{t_{j+1}}{\left(\tau -t_{j}\right)\left(t_{n+1}-\tau \right)}^{\sigma -1}d\tau \right), \end{array} \end{array}$$

(150) $$\begin{array}{c} \begin{array}{c} R_{n+1}=R_{0}+\frac{\left(1-\sigma \right)}{\text{ABC}\left(\sigma \right)}\left\{-aR\left(t_{n}\right)+edS\left(t_{n}\right)\right\}\\ +\frac{\sigma }{\Gamma \left(\sigma \right)\times \text{ABC}\left(\sigma \right)}\overset{n}{\underset{j=0}{\sum }}\left(\frac{\left\{-aR_{j}+edS_{j}\right\}}{h}\right.\\ \times \int_{t_{j}}^{t_{j+1}}\left(\tau -t_{j-1}\right){\left(t_{n+1}-\tau \right)}^{\sigma -1}d\tau \\ \left.-\frac{\left\{-aR_{j-1}+edS_{j-1}\right\}}{h}\times \int_{t_{j}}^{t_{j+1}}\left(\tau -t_{j}\right){\left(t_{n+1}-\tau \right)}^{\sigma -1}d\tau \right). \end{array} \end{array}$$

By using equations (133) and (144), we get

(151) $$\begin{array}{c} \begin{array}{c} P_{n+1}=P_{0}+\frac{\left(1-\sigma \right)}{\text{ABC}\left(\sigma \right)}\left\{\text{a}-aP\left(t_{n}\right)-bP\left(t_{n}\right)S\left(t_{n}\right)\right\}\\ +\frac{\sigma }{\text{ABC}\left(\sigma \right)}\overset{n}{\underset{j=0}{\sum }}\left(\frac{h^{\sigma }\left\{\text{a}-aP_{j}-bP_{j}S_{j}\right\}}{\Gamma \left(\sigma +2\right)}\times \left\{p_{1}p_{2}-p_{3}p_{4}\right\}\right.\\ \left.-\frac{h^{\sigma }\left\{\text{a}-aP_{j-1}-bP_{j-1}S_{j-1}\right\}}{\Gamma \left(\sigma +2\right)}\times \left\{p_{5}-p_{3}p_{6}\right\}\right), \end{array} \end{array}$$

(152) $$\begin{array}{c} \begin{array}{c} L_{n+1}=L_{0}+\frac{\left(1-\sigma \right)}{\text{ABC}\left(\sigma \right)}\left\{-aL\left(t_{n}\right)+bP\left(t_{n}\right)L\left(t_{n}\right)-cL\left(t_{n}\right)S\left(t_{n}\right)\right\}\\ +\frac{\sigma }{\text{ABC}\left(\sigma \right)}\overset{n}{\underset{j=0}{\sum }}\left(\frac{h^{\sigma }\left\{-aL_{j}+bP_{j}L_{j}-cL_{j}S_{j}\right\}}{\Gamma \left(\sigma +2\right)}\times \left\{p_{1}p_{2}-p_{3}p_{4}\right\}\right.\\ \left.-\frac{h^{\sigma }\left\{-aL_{j-1}+bP_{j-1}L_{j-1}-cL_{j-1}S_{j-1}\right\}}{\Gamma \left(\sigma +2\right)}\times \left\{p_{5}-p_{3}p_{6}\right\}\right), \end{array} \end{array}$$

(153) $$\begin{array}{c} \begin{array}{c} S_{n+1}=S_{0}+\frac{\left(1-\sigma \right)}{\text{ABC}\left(\sigma \right)}\left\{-\left(a+d\right)S\left(t_{n}\right)+cL\left(t_{n}\right)S\left(t_{n}\right)+fQ\left(t_{n}\right)\right\}\\ +\frac{\sigma }{\text{ABC}\left(\sigma \right)}\overset{n}{\underset{j=0}{\sum }}\left(\frac{h^{\sigma }\left\{-\left(a+d\right)S_{j}+cL_{j}S_{j}+fQ_{j}\right\}}{\Gamma \left(\sigma +2\right)}\times \left\{p_{1}p_{2}-p_{3}p_{4}\right\}\right.\\ \left.-\frac{h^{\sigma }\left\{-\left(a+d\right)S_{j-1}+cL_{j-1}S_{j-1}+fQ_{j-1}\right\}}{\Gamma \left(\sigma +2\right)}\times \left\{p_{5}-p_{3}p_{6}\right\}\right), \end{array} \end{array}$$

(154) $$\begin{array}{c} \begin{array}{c} Q_{n+1}=Q_{0}+\frac{\left(1-\sigma \right)}{\text{ABC}\left(\sigma \right)}\left\{-\left(a+f\right)Q\left(t_{n}\right)+d\left(1-e\right)S\left(t_{n}\right)\right\}\\ +\frac{\sigma }{\text{ABC}\left(\sigma \right)}\overset{n}{\underset{j=0}{\sum }}\left(\frac{h^{\sigma }\left\{-\left(a+f\right)Q_{j}+d\left(1-e\right)S_{j}\right\}}{\Gamma \left(\sigma +2\right)}\times \left\{p_{1}p_{2}-p_{3}p_{4}\right\}\right.\\ \left.-\frac{h^{\sigma }\left\{-\left(a+f\right)Q_{j-1}+d\left(1-e\right)S_{j-1}\right\}}{\Gamma \left(\sigma +2\right)}\times \left\{p_{5}-p_{3}p_{6}\right\}\right), \end{array} \end{array}$$

(155) $$\begin{array}{c} \begin{array}{c} R_{n+1}=R_{0}+\frac{\left(1-\sigma \right)}{\text{ABC}\left(\sigma \right)}\left\{-aR\left(t_{n}\right)+edS\left(t_{n}\right)\right\}\\ +\frac{\sigma }{\text{ABC}\left(\sigma \right)}\overset{n}{\underset{j=0}{\sum }}\left(\frac{h^{\sigma }\left\{-aR_{j}+edS_{j}\right\}}{\Gamma \left(\sigma +2\right)}\times \left\{p_{1}p_{2}-p_{3}p_{4}\right\}\right.\\ \left.-\frac{h^{\sigma }\left\{-aR_{j-1}+edS_{j-1}\right\}}{\Gamma \left(\sigma +2\right)}\times \left\{p_{5}-p_{3}p_{6}\right\}\right). \end{array} \end{array}$$

where

(156) $$\begin{array}{c} p_{1}={\left(m+1-j\right)}^{\sigma }, \end{array}$$

(157) $$\begin{array}{c} p_{2}=\left(m-j+2+\sigma \right), \end{array}$$

(158) $$\begin{array}{c} p_{3}={\left(m-j\right)}^{\sigma }, \end{array}$$

(159) $$\begin{array}{c} p_{4}=\left(m-j+2+2\sigma \right), \end{array}$$

(160) $$\begin{array}{c} p_{5}={\left(m+1-j\right)}^{\sigma +1}, \end{array}$$

(161) $$\begin{array}{c} p_{6}=\left(m-j+1+\sigma \right). \end{array}$$

The article "Analysis and Simulation of Fractional Order Smoking Epidemic Model" was published in 2022. Journal: Comput Math Methods Med.

## 7. Numerical Results and Discussion

A mathematical study of the nonlinear epidemic model of smoking has been presented. For checking of parameters effects on smoking dynamical model, relatively some numerical simulations according to the value of the parameters are accomplished to confirm the effect of the fractional derivative on the different compartments. We got mathematical consequences of the model for different fractional values with the help of the ATM. If we note the impacts of variables on the dynamics of the model of fractional order, the end-time value of the given parameter can be observed in various numerical ways. We can observe that the results of fractional value are more accurate as compared to classical derivatives. Desired results can be achieved to analyze the epidemic that occurs due to smoking. The graphs of the approximate solutions are given in Figures 1–5 against different fractional-order *α*. *P*(*t*) and *R*(*t*) start decreasing by decreasing the fractional values while *L*(*t*), *S*(*t*), and *Q*(*t*) start increasing by decreasing fractional values which can be easily observed in Figures 1–5. When the fractional values decrease then the behavior approaches steady-state in all figures, which shows that the solution will be more effective by decreasing the fractional values.

## 8. Conclusion

The advanced numerical scheme of fractional differential equation has been investigated in this article for smoking model by using ATM. With the help of fixed point theory uniqueness and stability of the smoking, the model has been examined. System is analyzed qualitatively to verify the steady state position of the dynamic. Proposed system is analyzed locally; also, global stability has been made using first derivative of Lyapunov. The arbitrary derivative of fractional order has been taken in ATM with no singular kernel. Effective results are obtained for the proposed model. Also discussed some theoretical results and proved the efficiency of the proposed techniques. Numerical simulations are carried out to check the actual behavior of the dynamic using the advanced ATM. These results will be helpful to understand further analysis and to control different outbreak caused by smoking.

## Figures and Tables

**Figure 1:** Simulation of *P*(*t*) with ABC fractional-order scheme.

**Figure 2:** Simulation of *L*(*t*) with ABC fractional-order scheme.

**Figure 3:** Simulation of S(t) with ABC fractional-order scheme.

**Figure 4:** Simulation of *Q*(*t*) with ABC fractional-order scheme.

**Figure 5:** Simulation of *R*(*t*) with ABC fractional-order scheme.

## Data Availability

No data were used to support this study.
